The article "Comparison of predictions of daily evapotranspiration based on climate variables using different data mining and empirical methods in various climates of Iran" was retracted in 2026. Reasons: unreliable results or conclusions; concerns about the citations.

# Comparison of predictions of daily evapotranspiration based on climate variables using different data mining and empirical methods in various climates of Iran

**DOI:** 10.1016/j.heliyon.2023.e13245

**Published:** 2023-01-28

**Authors:** Saeed Sharafi, Mehdi Mohammadi Ghaleni, Miklas Scholz

**Affiliations:** a Department of Environment Science and Engineering, Arak University, Arak, Iran; b Department of Water Science and Engineering, Arak University, Arak, Iran; c Department of Asset Management und Strategic Planning, Oldenburgisch‐Ostfriesischer Wasserverband, Georgstraße 4, 26919, Brake (Unterweser), Germany; d Department of Civil Engineering Science, School of Civil Engineering and the Built Environment, University of Johannesburg, Kingsway Campus, PO Box 524, Aukland Park 2006, Johannesburg, South Africa; e Directorate of Engineering the Future, School of Science, Engineering and Environment, The University of Salford, Newton Building, Greater Manchester, M5 4WT, United Kingdom; f Department of Town Planning, Engineering Networks and Systems, South Ural State University (National Research University), 76, Lenin prospekt, Chelyabinsk 454080, Russian Federation

**Keywords:** Aridity index, Artificial intelligence technique, Environmental software evaluation, Machine learning, Scatter index, Water resources management

## Abstract

To accurately manage water resources, a precise prediction of reference evapotranspiration (ET_ref_) is necessary. The best empirical equations to determine ET_ref_ are usually the temperature-based Baier and Robertson (BARO), the radiation-based Jensen and Haise (JEHA), and the mass transfer-based Penman (PENM) ones. Two machine learning (ML) models were used: least squares support vector regression (LSSVR) and ANFIS optimized using the particle swarm optimization algorithm (ANFPSO). These models were applied to the daily ET_ref_ at 100 synoptic stations for different climates of Iran. Performance of studied models was evaluated by the correlation coefficient (R), coefficient of determination (R^2^), mean absolute error (MAE), root mean square error (RMSE), scatter index (SI) and the Nash-Sutcliffe efficiency (NSE). The combination-based ML models (LSSVR4 and ANFPSO4) had the lowest error (RMSE = 0.34–2.85 mm d^−1^) and the best correlation (R = 0.66–0.99). The temperature-based empirical relationships had more precision than the radiation- and mass transfer-based empirical equations.

## 1 Introduction

Arid regions of the world are more sensitive to climate change and variability concerning hydroclimatic conditions. The uptake of water resources has considerably increased, because of increasing global population and average human water withdrawals per capita [1,2]. To achieve water resource sustainability, accurate ET_ref_ estimation is necessary. ET_ref_ estimation is a non-linear relationship that is a function of several meteorological variables [[3], [4], [5], [6], [7], [8], [9], [10], [11]].

The article "Comparison of predictions of daily evapotranspiration based on climate variables using different data mining and empirical methods in various climates of Iran" was retracted in 2026. Reasons: unreliable results or conclusions; concerns about the citations.

A precise determination of ET_ref_ can be performed with a lysimeter station. However, establishing these stations can be expensive, particularly in developing countries. The Penman-Monteith equation based on FAO_56_ (PM-FAO_56_) has typically been used as a semi-empirical equation for prediction of ET_ref_ [[12], [13], [14], [15]]. In spite of the acceptance of the PM-FAO_56_ equation, it requires full datasets of climatic variables. However, such data are often not available and/or are incomplete. On the other hand, the calculation of ET_ref_ may be considered as simulating a non-linear association between ET_ref_ and a large number of climatic variables [16]. Therefore, researchers studied and evaluated so far ET_ref_ models in various climates [15,[17], [18], [19], [20]]. The empirical models are usually divided into four categories: models based on temperature, radiation and mass transfer as well as a combination of various models [6,14,[21], [22], [23]].

Furthermore, different algorithms and methods have been so far developed for the calculation of ET_ref_, including artificial neural network (ANN) [[24], [25], [26], [27], [28]], SVM [[29], [30], [31]], ANFIS [[32], [33], [34], [35], [36], [37], [38], [39]], multiple layer perceptron (MLP; [[40], [41], [42]]), generalized regression neural networks (GNN; [43]), extreme learning machine (ELM; [34,35,[44], [45], [46], [47], [48]]). Among the methods listed, numerous ET_ref_ models have been evaluated by researchers using ELM methods. ELM methods are theoretically alternatives, because they generate simple equations and use a more limited number of climatic variables than the PM-FAO_56_ model. These methods use LSSVR, ANN, PSO, GA and GEP and are utilized by many researchers [19,47,[49], [50], [51], [52]]. Of these models, LSSVR and ANFPSO have been found to generate more accurate results.

Chen [25] applied LSSVR and ANN models for the prediction of daily ET_ref_ in a semi-arid climate. By comparing the results with MLR, he concluded that the ANN model, which uses all climatic variables as input, has the best performance. Kisi et al. [53] modeled the values of mean monthly ET_ref_ for Iran using data-driven methods of ANN, GEP, ANFIS-grid partitioning (ANFIS-GP) and ANFIS-subtractive clustering (ANFIS-SC). They concluded that ANFIS-GP has the best performance among the studied methods. In India Patil and Deka [54] estimated weekly ET_ref_ and compared the performance of ANN, LSSVM and ELM methods. The ELM provided better results for the estimation of ET_ref_ than the ANN and SVM methods. Zhu et al. [47] evaluated the PSO algorithm to obtain the parameters of the ELM method. Afterwards, a hybrid PSO-ELM model was suggested to calculate approximate daily ET_ref_ for the arid climate of China. They confirmed that the PSO-ELM method was more reliable than other ELM models and empirical equations, and thus suggested its use to compute daily ET_ref_.

The article "Comparison of predictions of daily evapotranspiration based on climate variables using different data mining and empirical methods in various climates of Iran" was retracted in 2026. Reasons: unreliable results or conclusions; concerns about the citations.

The main novelty of the research is the comprehensive comparison of data mining models with the most appropriate empirical equations [14] to predict the daily potential evapotranspiration across different climates. Furthermore, Iran has a long dry season (six to eight months) with rainfall amounts less than 5% of the total precipitation [6,55].

The main objectives of the present study are as follows: (i) to compare the correctness of different ML models (LSSVR and ANFPSO) and empirical equations (BARO, JEHA and PENM) in daily ET_ref_ estimation; (ii) to evaluate models with different combinations of climate inputs (temperature-, radiation- and mass transfer-based as well as combination-based); and (iii) to recommend optimal ML models to predict the daily ET_ref_ using limited input data for the various climates across Iran. Moreover, two approaches were pursued to assess the performance of the recommended methods for calculating ET_ref_: (a) suggested models were tested and trained for 100 synoptic stations; and (b) the synoptic stations were divided into four climate classes using the UNESCO aridity index with their mean climatic traits. The flowchart of the research undertaken is present in Fig. 1.

**Fig. 1:** Outline of the research.

## 2 Materials and methods

### 2.1 Case study and associated data

The meteorological data of 100 synoptic stations across Iran were used. The station locations are presented in Fig. 2. The meteorological data were obtained from IRIMO and included mean, maximum (T_max_) and minimum (T_min_) air temperatures, precipitation, relative humidity, wind speed and solar radiation for a period of 33 years (1987–2019). Altitude differences among the stations ranged from 26 m below sea level at Bandar Anzali station to 2465 m above sea level at Abali station. A double-mass curve analysis was conducted to evaluate the quality of the meteorological data [56]. Missing data were replaced by the means between the corresponding data for the previous and following years. The Angstrom equation was used to fill the solar radiation gaps [57] when the correlation was more than 0.8 at the 95% confidence level. First of all, solar radiation meeting the land (R_n_, MJ m^−2^ d^−1^) was determined above the earth's atmosphere for each day linked to the corresponding latitude and longitude as well as the solar constant [57]. Then, equation (1) was used to calculate the value of R_s_.

(1) $$Rs=K_{Rs}\times \left(1+2.7\times 10^{-5}\times Alt\right)\times {\left(T_{\max}-T_{\min}\right)}^{0.5}\times R_{n}$$

where Alt is altitude (m); and K_Rs_ is the empirical constant, considered equal to 0.16 [6] Precipitation values in Iran are also very diverse so that the average annual precipitation during the study varied from 52.6 mm at Zabol station to 1694.7 mm at Anzali station. The average annual ET_ref_ calculated with the PM-FAO_56_ equation varied from about 800 mm at Anzali station to about 5040 mm at Jask station.

The article "Comparison of predictions of daily evapotranspiration based on climate variables using different data mining and empirical methods in various climates of Iran" was retracted in 2026. Reasons: unreliable results or conclusions; concerns about the citations.

**Fig. 2:** Location and climate class of synoptic stations based on the ratio of precipitation to ET_ref_.

Based on meteorological parameters, climates in Iran range from arid to humid. The UNESCO aridity index was applied for temperature-based and precipitation-based climate classifications and is calculated using the values of P and ET_ref_ (Eq. (2)). According to this classification, climate can be divided according to these categories: hyper-arid (AI<0.03), arid (0.03 < AI<0.20), semi-arid (0.20 < AI<0.50) and humid (AI>0.50) [[58], [59], [60]]. The AI_UNESCO_ varied from 0.01 at Zabol station to 2.12 at Anzali station (Eq. (2)).

(2) $$AI_{UNESCO}=\frac{P}{ET_{ref}}\times 100$$

According to the AI_UNESCO_, 10 stations were located in hyper-arid climate, 48 stations were situated in arid climate, 30 stations were located in semi-arid climate and 12 stations can be found in humid climate (Table 1). In general, the central and southeastern regions of Iran have a hyper-arid climate, and the northeastern, southern and southwestern regions have an arid climate. The western and northwestern regions of Iran have a semi-arid climate. The Caspian Sea region has a humid climate (Fig. 2).

**Table 1:** Stations according to climate classification.

Climate Classification	Stations
Hyper-arid	Zabol, Yazd, Bam, Anar, Jask, Khorobiabank, Siri, Tabass, Chabahar and Abumusa
Arid	Iranshahr, Kerman, Nehbandan, Bandar Lengeh, Kashan, Garmsar, Zahedan, Khash, Kish, Qom, Saravan, Bandar Abbas, East Isfahan, Abadan, Sirjan, Bushehr, Ferdows, Shahr Babak, costal Bushehr, Shahroud, Minab, Birjand, Ghaen, Semnan, Gonabad, Bostan, Isfahan, Ahwaz, Sabzevar, Omidieh, Karaj, Kashmar, Abadeh, Golmakan, Tehran, Fassa, Mashhad, Ramhormoz, Safiabad, Shiraz, Torbat-e Heydarieh, Sarakhs, Sarpolzahab, Ghochan, Masjedsoleiman, Bojnord and Mianeh
Semi-arid	Jolfa, Sarab, Tabriz, Urmia, Arak, Hamedan Nozheh, Hamedan Airport, Parsabad, Maragheh, Khorramdareh, Ahar, Makoo, Shahrekord, Qazvin, Ardabil, Sanandaj, Takab, Bijar, Kangavar, Zanjan, Saqez, Mahabad, Kermanshah, Khalkhal, Aligoodarz, Islamabad, Dogonbadan, Khorramabad, Ilam and Ravansar
Humid	Abali, Gorgan, Piranshahr, Gharakhil, Sardasht, Babolsar, Koohrang, Rasht, Rasht and Anzali

Fig. 3 illustrates the range of changes of the four parameters T_min_, T_max_, P and ET_ref_. The lowest and highest values of T_min_ were recorded in semi-arid and hyper-arid climates, respectively (Fig. 3a). T_max_ values from arid to humid climates show a decreasing trend (Fig. 3b). Fig. 3c shows the increasing trend of P from hyper-arid to humid climates. The decreasing trend of annual ET_ref_ values is also shown in Fig. 3d.

The article "Comparison of predictions of daily evapotranspiration based on climate variables using different data mining and empirical methods in various climates of Iran" was retracted in 2026. Reasons: unreliable results or conclusions; concerns about the citations.

**Fig. 3:** Boxplots showing meteorological variables of (a) T_min_; (b) T_max_; P; and (d) ET_ref_ for different climates of Iran.

### 2.2 Empirical ET_ref_ relationships

According to the importance and category of input climatic parameters applied by empirical equations to compute the daily ET_ref_, all models were categorized subject to these four classes: temperature-based (BARO equation), solar radiation–based (JEHA equation), mass transfer–based (PENM equation) and combination-based (PM-FAO_56_). These empirical equations were introduced by Sharafi and Mohammadi Ghaleni [14] and gave good results in each category and are therefore recommended for estimating ET_ref_ in different climates of Iran. To compare the results of different models, the PM-FAO_56_ equation was calculated for all stations. The empirical equations are given below (Eqs. (3), (4), (5), (6))):

BARO (Baier and Robertson [61])

(3) $$ET_{ref}=0.109\times \left(R_{a}/\lambda \right)+0.157T_{\max}+0.158\left(T_{\max}-T_{\min}\right)-5.39$$

JEHA (Jensen and Haise [62])

(4) $$ET_{ref}=\left(0.025T_{mean}+0.08\right)R_{s}/\lambda$$

PENM (Penman [63])

(5) $$ET_{ref}=\left(2.625+0.000479u_{2}\right)\left(e_{s}-e_{a}\right)$$

PM-FAO56 (Allen et al. [57])

(6) $$ET_{ref}=\frac{0.408\Delta \left(R_{n}-G\right)+\gamma \left[900/\left(T_{mean}+273\right)\right]u_{2}\left(e_{s}-e_{a}\right)}{\Delta +\gamma \left(1+0.34u_{2}\right)}$$

where Δ is the slope of the saturation vapor pressure function (kPa °C^−1^), R_n_ is the net radiation (MJ m^−2^ d^−1^), G is the soil heat flux density (MJ m^−2^ d^−1^), γ is the psychometric constant (kPa °C^−1^), T_mean, max and min_ are the mean, maximum and minimum daily temperatures (°C) in this order, u_2_ is the wind speed (m s^−1^) measured at a height of 2 m, R_a_ is the extraterrestrial radiation (MJ m^−2^ d^−1^), ʎ is the latent heat of vaporization (MJ kg^−1^), RH is the mean relative humidity (%), R_s_ is the solar radiation (MJ m^−2^ d^−1^), e_s_ is the saturation vapor pressure (kPa), e_a_ is the actual vapor pressure (k Pa), and (e_s_-e_a_) is the saturation vapor pressure deficit (kPa).

The article "Comparison of predictions of daily evapotranspiration based on climate variables using different data mining and empirical methods in various climates of Iran" was retracted in 2026. Reasons: unreliable results or conclusions; concerns about the citations.

### 2.3 ML models

#### 2.3.1 LSSVR algorithm

The least squares support vector regression (LSSVR [64]) was introduced for classification (discrete) and regression (real) challenges. According to the supervised learning method, a concept known as structural risk minimization is utilized to minimize the error of the model, whereas other methodologies (e.g. ANN) apply the principles of Empirical Risk Minimization [65]. In LSSVR, data are linearly separated and a regression line with the greatest confidence level is determined. Convex Quadratic Programming is used to solve the optimal line equations, which makes the problem complex and time-consuming [66]. Thus, solving large-scale challenges using this methodology entails high computational costs and makes the algorithm more complex. However, LSSVR converts the non-linear relationship between inputs and outputs to a linear relationship. The advantages of LSSVR include high precision and accuracy, low complexity, mathematical tractability and speed. One of the factors affecting the LSSVR accuracy is the selection of an appropriate Kernel Function [67].

#### 2.3.2 ANFPSO algorithm

In the ANFPSO model, ET_ref_ prediction has been performed using two models. ANFIS has been optimized using the particle swarm optimization algorithm. The ANFIS model has five layers including membership, fuzzy, normalization, diffusion and output layers. Fuzzy input variables have input membership functions (membership rules), while output membership functions and diffused output are the outputs of the first to fifth layers of the ANFIS model, respectively [68].

In this paper, the ANFIS model has been presented. This model is based on five input layers and the Gaussian membership function. The Levenberg–Marquardt algorithm was used to teach the ANFIS model. In the combined model ANFPSO, the particle swarm optimization (PSO) algorithm has been used to teach the ANFIS model. In other words, in this hybrid model, the weights of membership functions in the ANFIS model are optimized by the PSO algorithm to minimize the difference between measured and predicted ET_ref_. Also, different meta-heuristic methods can be used to train the standard mathematical ML.

The PM-FAO_56_ was calculated as the target ET_ref_ and these four groups of empirical ML models were selected: combination-based, radiation-based, temperature-based and mass transfer based. Table 2 showed the input variables for each model.

The article "Comparison of predictions of daily evapotranspiration based on climate variables using different data mining and empirical methods in various climates of Iran" was retracted in 2026. Reasons: unreliable results or conclusions; concerns about the citations.

**Table 2:** Input variables for ML and empirical equation models.

Type model	Model category	Input variables	Model name
1	Temperature-based	T_max_, T_min_ and R_a_	LSSVR1
			ANFPSO1
			BARO
2	Radiation-based	T_max_, T_min_, R_a_ and R_s_	LSSVR2
			ANFPSO2
			JEHA
3	Mass transfer-based	T_max_, T_min_, RH and U_2_	LSSVR3
			ANFPSO3
			PENM
4	Combination-based	T_max_, T_min_, R_a_, R_s_, RH and U_2_	LSSVR4
			ANFPSO4
			PM-FAO_56_

### 2.4 Evaluation performance criteria

In this study, the number of eight statistical criteria were evaluated for each synoptic station: coefficient of determination (R^2^), mean absolute error (MAE), the root mean square error (RMSE), the average percentage error (APE), Nash-Sutcliffe Efficiency (NSE), the index of agreement (D) and the scatter index (SI). The perfect value for MAE, RMSE, SI, and MAE indices is zero, and for NSE and R^2^ is unity. Li et al. [69] characterized the range of SI for the precision of the models as follows: excellent (SI < 0.1), good (0.1 < SI < 0.2), fair (0.2 < SI < 0.3) and poor (SI > 0.3). These criteria were applied, previously [6,14,21,70]. They are commonly used to assess the results of empirical equations as well as LSSVR and ANFPSO models with PM-FAO_56_ on the basis of Eqs. (7), (8), (9), (10), (11), (12).

Correlation coefficient (R) (Ma and Iqbal [71])

(7) $$R=\frac{\sum_{N}^{i=1}\left(ET_{ref_{i}}^{P{M_{FAO}}_{56}}-{\bar{ET}}_{ref}^{P{M_{FAO}}_{56}}\right)\left(ET_{ref_{i}}^{\mathrm{mod}\;el}-{\bar{ET}}_{ref}^{\mathrm{mod}\;el}\right)}{\sqrt{\left[\sum_{i=1}^{N}{\left(ET_{ref_{i}}^{P{M_{FAO}}_{56}}-{\bar{ET}}_{ref}^{P{{M_{F}}_{AO}}_{56}}\right)}^{2}\right]\left[\sum_{i=1}^{N}{\left(ET_{ref_{i}}^{\mathrm{mod}\;el}-{\bar{ET}}_{ref}^{\mathrm{mod}\;el}\right)}^{2}\right]}}$$

Mean Absolute Error (MAE) (M44a and Iqbal [71])

(8) $$MAE=\frac{1}{N}\sum_{N}^{i=1}\left|ET_{Ref_{i}}^{\mathrm{mod}\;el}-ET_{Ref_{i}}^{PMF56}\right|$$

Nash-Sutcliffe Efficiency (NSE) (Ferreira and da Cunha [49])

(9) $$NSE=1-\left[\frac{\sum_{N}^{i=1}{\left(ET_{Ref_{i}}^{PMF56}-ET_{Ref_{i}}^{\mathrm{mod}\;el}\right)}^{2}}{\sum_{i=1}^{N}{\left(ET_{Ref_{i}}^{PMF56}-{\bar{ET}}_{Ref}^{PMF56}\right)}^{2}}\right]$$

Root mean square error (RMSE) (Ma and Iqbal [71])

(10) $$RMSE=\sqrt{\frac{1}{N}\sum_{i=1}^{N}{\left(ET_{ref_{i}}^{\mathrm{mod}\;el}-ET_{ref_{i}}^{PM_{{{}_{F}}_{56}}}\right)}^{2}}$$

Coefficient of determination (R^2^) (Ma and Iqbal [71])

(11) $$R^{2}={\left[\frac{\sum_{N}^{i=1}\left(ET_{ref_{i}}^{P{M_{FAO}}_{56}}-{\bar{ET}}_{ref}^{P{M_{FAO}}_{56}}\right)\left(ET_{ref_{i}}^{\mathrm{mod}\;el}-{\bar{ET}}_{ref}^{\mathrm{mod}\;el}\right)}{\sqrt{\left[\sum_{i=1}^{N}{\left(ET_{ref_{i}}^{P{M_{FAO}}_{56}}-{\bar{ET}}_{ref}^{P{{M_{F}}_{AO}}_{56}}\right)}^{2}\right]\left[\sum_{i=1}^{N}{\left(ET_{ref_{i}}^{\mathrm{mod}\;el}-{\bar{ET}}_{ref}^{\mathrm{mod}\;el}\right)}^{2}\right]}}\right]}^{2}$$

Scatter Index (SI) (Li et al. [69])

(12) $$SI=\frac{RMSE}{{\bar{ET}}_{ref}^{P{M_{FAO}}_{56}}}$$

where in Eqs. (7), (8), (9), (10), (11), (12), $ET_{ref_{i}}^{PM_{FAO56}}$ and $ET_{ref_{i}}^{\mathrm{mod}\;el}$ are the ET_ref_ based on PM-FAO_56_ and modeled ET_ref_, ${\bar{ET}}_{ref}^{P{M_{FAO}}_{56}}$ and ${\bar{ET}}_{ref}^{\mathrm{mod}\;el}$ are the mean values of ET_ref_ based on PM-FAO_56_ and modeled ET_ref_, and N is the number of datasets for 12,053 days.

The article "Comparison of predictions of daily evapotranspiration based on climate variables using different data mining and empirical methods in various climates of Iran" was retracted in 2026. Reasons: unreliable results or conclusions; concerns about the citations.

## 3 Results

Boxplots and mean values of performance metrics were used to evaluate R, MAE, NSE, RMSE, R^2^ and SI for each synoptic stations to analyze time series plots of predicted versus observed numbers and the behavior of models during the time period 1987–2019. The distribution of NSE values in space and SI mapping for all ML models and empirical equations listed are presented for each synoptic stations in Fig. 4, Fig. 5, Fig. 6, Fig. 7, respectively.

**Fig. 4:** Heat map for showing (a) correlation coefficients; and (b) mean absolute errors between ML models and empirical equations with PM-FAO_56_ in different climates of Iran.

**Fig. 5:** Time series plots and the distribution of NSE values in space for ML models and empirical equations for different Iranian climates.

**Fig. 6:** Residuals (error plot) of the four types of models for dailly ET_ref_ estimation concerning various climates: (a) hyper-arid; (b) arid; (c) semi-arid; and (d) humid climates of Iran.

**Fig. 7:** Spatial patterns of SI for (a) LSSVR models; (b) ANFPSO models; and (c) empirical equations for 100 synoptic stations of Iran.

Fig. 4 illustrates the heating map of the R and MAE values according to ML models and the empirical equations. The mean R for ML models (LSSVR1-4 and ANFPSO1-4) and empirical equations (BARO, HEHA and PENM) for all studied stations are 0.83 and 0.69, correspondingly (Fig. 4a). The mean MAE values for the studied stations for intelligent models and empirical equations were 0.76 and 1.89 mm d^−1^, respectively (Fig. 4b). These results show that the ML models are more accurate than the empirical equations based on R and MAE results.

Mean R and MAE for temperature-based (LSSVR1, ANFPSO1 and BARO), radiation-based (LSSVR2, ANFPSO2 and JEHA), mass transfer-based (LSSVR3, ANFPSO3 and PENM) and combination-based (LSSV4 and ANFPSO4) models were 0.82, 0.75, 0.76, 0.86 and 0.87, 1.29, 1.33, 0.62 in this order. In other words, the highest and lowest accuracy in ET_ref_ estimation were related to the ML models (R = 0.86 and MAE = 0.62 mm d^−1^) and the mass transfer-based models (R = 0.76 and MAE = 1.33 mm d^−1^).

The article "Comparison of predictions of daily evapotranspiration based on climate variables using different data mining and empirical methods in various climates of Iran" was retracted in 2026. Reasons: unreliable results or conclusions; concerns about the citations.

Comparisons between climates showed that the average R of 11 ML models and empirical equations for stations located in hyper-arid, arid, semi-arid and humid climates are 0.69, 0.79, 0.86 and 0.69, correspondingly. The mean MAE in all studied models from hyper-arid to humid climates were 2.94, 1.18, 0.49 and 0.47 mm d^−1^, respectively. This shows that there was no difference between selected stations in each climate and that the climate classification based on AI_UNESCO_ values was suitable. ML models and empirical equations in semi-arid (R = 0.86 and MAE = 0.49 mm d^−1^) and hyper-arid (R = 0.69 and MAE = 2.94 mm d^−1^) climates had the highest and lowest accuracy in estimating daily ET_ref_, respectively.

### 3.1 Temperature-based models

The application of classical ML models to evaluate ET_ref_ has recently attracted the attention of many researchers, and it has been confirmed that ML models provide better results than empirical equations [5,72]. The performance of recommended models in the temperature-based method is demonstrated in Fig. 4. The average value of R for temperature-based models in all stations studied for BARO, ANFPSO1 and LSSVR1 models are 0.85, 0.80 and 0.81, respectively (Fig. 4a). The mean R of BARO were 0.043 and 0.051 higher than those of LSSVR1 and ANFPSO1, and the mean MAE of LSSVR1 were 0.028 and 0.19 mm d^−1^ lower than those of ANFPSO1 and BARO (Fig. 4b).

According to the findings, there was no significant difference between the LSSVR1 and ANFPSO1 models in terms of RMSE, but the LSSVR1 model outperformed the ANFPSO1 and BARO. These results demonstrate that temperature-based LSSVR1 achieved a higher precision when calculating ET_ref_ compared to the use of the BARO equation. In contrast, ANFPSO1 decreased the R^2^ by 0.089, and also decreased the RMSE, showing that the temperature-based LSSVR1 model slightly outperformed ET_ref_ (Table 3).

**Table 3:** RMSE and R^2^ criteria for different models in different climates.

Base	Model	Step	Hyper-arid		Arid		Semi-arid		Humid	
			RMSE	R^2^	RMSE	R^2^	RMSE	R^2^	RMSE	R^2^
Temperature	LSSVR1	All	2.95	0.53	1.14	0.67	0.43	0.78	0.44	0.51
		Train	2.86	0.55	1.10	0.70	0.42	0.82	0.43	0.53
		Test	3.16	0.50	1.23	0.63	0.46	0.74	0.47	0.48
	ANFPSO1	All	3.04	0.51	1.16	0.66	0.44	0.77	0.45	0.49
		Train	2.94	0.53	1.13	0.69	0.42	0.81	0.43	0.51
		Test	3.27	0.48	1.24	0.62	0.47	0.73	0.48	0.47
	BARO1	All	4.74	0.48	1.36	0.75	0.45	0.87	0.39	0.76
Radiation	LSSVR2	All	3.32	0.44	1.29	0.62	0.43	0.78	0.45	0.49
		Train	3.22	0.46	1.24	0.66	0.42	0.82	0.44	0.51
		Test	3.57	0.42	1.39	0.59	0.46	0.74	0.49	0.46
	ANFPSO2	All	3.35	0.43	1.30	0.61	0.44	0.77	0.46	0.48
		Train	3.25	0.45	1.26	0.65	0.42	0.81	0.44	0.50
		Test	3.59	0.41	1.39	0.58	0.47	0.73	0.49	0.45
	JEHA2	All	5.77	0.30	2.85	0.47	1.51	0.57	1.28	0.34
Mass transfer	LSSVR3	All	2.29	0.68	1.02	0.73	0.36	0.84	0.39	0.62
		Train	2.22	0.71	0.99	0.77	0.35	0.88	0.38	0.65
		Test	2.48	0.64	1.11	0.69	0.39	0.79	0.42	0.58
	ANFPSO3	All	2.29	0.68	1.02	0.73	0.36	0.84	0.39	0.62
		Train	2.22	0.71	0.99	0.77	0.35	0.88	0.38	0.65
		Test	2.48	0.64	1.11	0.69	0.39	0.79	0.42	0.58
	PENM3	All	9.18	0.23	3.50	0.37	1.59	0.46	1.48	0.08
Combination	LSSVR4	All	1.36	0.77	0.82	0.76	0.35	0.85	0.36	0.66
		Train	1.28	0.82	0.77	0.81	0.34	0.89	0.36	0.69
		Test	1.56	0.73	0.92	0.71	0.38	0.80	0.37	0.64
	ANFPSO4	All	2.63	0.58	1.03	0.70	0.40	0.80	0.40	0.60
		Train	2.54	0.61	0.99	0.74	0.39	0.85	0.38	0.63
		Test	2.85	0.55	1.10	0.66	0.43	0.76	0.43	0.57

The mean R of BARO is higher than the ANFPSO1 and LSSVR1 models. This relationship has a R of less than 0.40 for some hyper-arid and arid climate stations (e.g., Jask, Siri, Chabahar, Bandar Lengeh and Bushehr coastal). The lower accuracy of the BARO at synoptic stations in the islands and coastal strip of the Persian Gulf is related to the high RH of these regions and the more complex evapotranspiration process. This is confirmed when assessing the MAE values that were higher than 4 mm d^−1^ BARO at 5 stations of the Persian Gulf including Jask, Siri, Chabahar, Abumusa and Bushehr coastal stations. Even the LSSVR1 and ANFPSO1 models have MAE values higher than 4 mm d^−1^ for the two Jask and Siri stations in the hyper-arid climate, the mean of MAE in all stations studied for these models is lower than the BARO. In general, while the mean MAE values of BARO, ANFPSO1 and LSSVR1 models in hyper-arid climates were 3.6, 2.5 and 2.3 mm d^−1^, correspondingly, the mean MAE values of all temperature-based models in other arid, semi-arid and humid climates were below 1 mm d^−1^ (Fig. 4b).

The article "Comparison of predictions of daily evapotranspiration based on climate variables using different data mining and empirical methods in various climates of Iran" was retracted in 2026. Reasons: unreliable results or conclusions; concerns about the citations.

Negative values of the NSE coefficient for the BARO at Chabahar and Jask indicated that the temperature-based models were less accurate in estimating ET_ref_ at stations with high RH. The mean NSE coefficients for temperature-based models in hyper-arid, arid, semi-arid and humid climates are 0.47, 0.66, 0.75 and 0.54, respectively. This indicates lower accuracy of temperature-based models in stations with higher RH in hyper-arid and humid climates than in arid and semi-arid ones. Furthermore, in stations where high RH has a significant effect on the ET_ref_ process, temperature-based models cannot provide an accurate estimate of ET_ref_ (Fig. 5).

The range of estimated residual error for daily ET_ref_ computed over a cumulative 12,053 days for hyper-arid, arid, semi-arid and humid climates considering all temperature-based models were −5.6 to 14.7, −4.3 to 4.5, −2.3 to 2.6, and −2.2 to 1.8 mm d^−1^, respectively. The mean SI values in those climates were 0.33, 0.17, 0.14 and 0.17 in this order. Thus, it can be concluded that the lowest and highest accuracy of temperature-based models were in the hyper-arid and semi-arid climates, correspondingly (Fig. 6).

Commonly, BARO is one of the most precise empirical equations for computing ET_ref_ and is commonly used across Iran due to low requirements and its higher precision for weather data [14]. In most studies, the ML models also enhance the accuracy of computing ET_ref_ using temperature-based models [72,73]. Nevertheless, this study indicates that temperature-based LSSVR1 and ANFPSO1 models do not improve the precision when assessing ET_ref_, because the R^2^ values of these models had almost the same statistical results as BARO (Table 3). Tabari et al. [74] reported that the results attained with the ML models for ET_ref_ estimates were superior than those achieved with empirical equations. Ferreira et al. [49] found that the temperature-based ML with lower RMSE and better R^2^ values showed suitable results when compared to empirical methods. Feng et al. [75] also conveyed that the ML model had more accurate results than the empirical equations.

### 3.2 Radiation-based models

In the present study, JEHA was chosen as the best radiation-based empirical model [6] to conduct a comparison with the LSSVR2 and ANFPSO2 models. The results demonstrated that the recommended radiation-based LSSVR2 and ANFPSO2 models were significantly enhanced than the JEHA model. The performance of recommended models in the radiation-based method is demonstrated in Fig. 4. The mean R of radiation-based models in all stations studied for JEHA, ANFPSO2 and LSSVR2 models are 0.67, 0.78 and 0.79, respectively. The mean R of LSSVR2 was 0.12 and 0.01 higher than those of JEAH and ANFPSO2, and the mean MAE of LSSVR2 was 0.01 and 2.21 mm d^−1^ lower than those of ANFPSO2 and JEHA (Fig. 4b). Also, the mean NSE of LSSVR2 was 0.01 and 2.34 lower than those of ANFPSO2 and JEHA (Fig. 5). These results show no significant difference in the RMSE between LSSVR2 and ANFPSO2 models, but the LSSVR2 model outperformed both ANFPSO2 and JEHA. These results confirm that radiation-based LSSVR2 and ANFPSO2 reached greater precision when calculating ET_ref_ compared to methods using the JEHA empirical equation.

The MAE values were higher than 4 mm d^−1^ JEHA for eight stations: Jask, Siri, Chabahar, Abumusa, Kerman, Bushehr coastal, Safiabad and Torbate Heydarieh. However, the LSSVR2 and ANFPSO2 models have MAE values higher than 4 mm d^−1^ for the Jask, Siri and Abumusa stations in the hyper-arid climate. In general, the mean MAE values of the JEHA, ANFPSO2 and LSSVR2 models for the hyper-arid climates were 4.6, 2.7 and 2.6 mm d^−1^, correspondingly. These are the highest MAE values between climates of all radiation-based models (Fig. 4b).

The article "Comparison of predictions of daily evapotranspiration based on climate variables using different data mining and empirical methods in various climates of Iran" was retracted in 2026. Reasons: unreliable results or conclusions; concerns about the citations.

The mean NSE coefficients for ML radiation-based models in hyper-arid, arid, semi-arid and humid climates are 0.44, 0.62, 0.77 and 0.48 in this order. This indicates lower accuracy of radiation-based models in hyper-arid and humid climates than in arid and semi-arid climates (Fig. 5). The range of estimated residual error for daily ET_ref_ for all radiation-based models computed over a cumulative 12,053 days for hyper-arid, arid, semi-arid and humid climates were −5.3 to 11.5, −4.3 to 6.6, −2.3 to 4.9, −2.1 to 3.5 mm d^−1^, respectively. The mean SI values for these climates were 0.39, 0.26, 0.25 and 0.28, respectively. This shows that the lowest and highest precision of radiation-based models were in hyper-arid and semi-arid climates, respectively (Fig. 6).

Recent studies have confirmed that the variation in ET_ref_ can be clarified by temperature and solar radiation. Therefore, temperature-based empirical equations might be expected to provide better results for computing ET_ref_ [14,21,72]. Similarly, Feng et al. [75] also found that ML models had a higher accuracy for modeling ET_ref_ than the empirical models in China. Researchers [5] assessed the performance of SVR coupled with the whale optimization algorithm and the empirical equations for predicting ET_ref_ in Iranian hyper-arid, arid and semi-arid climates and found that SVR coupled with the whale optimization algorithm had a better performance than empirical models.

### 3.3 Mass transfer-based models

The different model performances for the mass transfer-based method are shown in Fig. 4. The mean R of the mass transfer-based models for the entire stations studied for the PENM, ANFPSO3 and LSSVR3 models are 0.45, 0.81 and 0.82, respectively. The mean R of LSSVR3 was 0.38 and 0.01 higher than those of PENM and ANFPSO3, and the mean MAE of LSSVR3 were 0.01 and 5.39 mm d^−1^ lower than those of ANFPSO3 and PENM (Fig. 4b). These results show that there was no significant difference in the RMSE between LSSVR3 and ANFPSO3 models, but the LSSVR3 model outperformed the ANFPSO3 and PENM. The results confirm that mass transfer-based LSSVR3 and ANFPSO3 achieved greater precision when calculating ET_ref_ than the PENM empirical equation (Table 3).

The MAE values were higher than 4 mm d^−1^ PENM for 21 stations. The LSSVR3 and ANFPSO3 models have MAE values lower than 4 mm d^−1^ for all stations in various climates. In general, the mean MAE values for the PENM, ANFPSO3 and LSSVR3 models applied to hyper-arid climates were 7.24, 1.85 and 1.84 mm d^−1^, respectively. Those are the highest MAE values of all mass transfer-based models between climates. The mean NSE coefficients for ML radiation-based models in hyper-arid, arid, semi-arid and humid climates were 0.68, 0.73, 0.84 and 0.62 in this order. This indicates lower accuracy of mass transfer-based models for humid climates compared to arid and semi-arid ones (Fig. 4b).

The article "Comparison of predictions of daily evapotranspiration based on climate variables using different data mining and empirical methods in various climates of Iran" was retracted in 2026. Reasons: unreliable results or conclusions; concerns about the citations.

The range of estimated residual error for daily ET_ref_ for all radiation-based models computed over a cumulative 12,053 days for hyper-arid, arid, semi-arid and humid climates were −6.1 to 18.7, −2.5 to 8.8, −1.3 to 6.5 and −1.3 to 3.8 mm d^−1^, respectively. The mean SI numbers for those climates were 0.44, 0.25, 0.24 and 0.30, respectively. Thus, it can be concluded that the lowest and highest accuracy of radiation-based models were in hyper-arid and semi-arid climates, respectively (Fig. 6).

Adding RH as input to mass transfer-based ML models significantly (p < 0.05) enhanced the accuracy of computing ET_ref_ when compared to temperature-based ML models. This finding compares well with those reported by Kiafar et al. [76], confirming higher accuracies in calculating ETref compared to the application of empirical equations. It is reasonable that the mass transfer-based empirical equations do not use extraterrestrial radiation as the input, whereas the radiation-based equations do. Chen et al. [77] confirmed that the accuracy of the ML models in comparison to the temperature-based and radiation-based models was enhanced by adding the RH trait. The reason for this result was that feeding more data to the ML models usually improves their precision in calculating ET_ref_.

### 3.4 Combination-based models

The levels of precision concerning the ML models and the PM-FAO56 equation are very common when ETref modeling is more complex [19,78]. The performance of the recommended models in the combination-based method is shown in Fig. 4. The mean R of the combination-based models for all stations studied for the ANFPSO4 and LSSVR4 models is 0.84 and 0.88, respectively. The mean R of LSSVR4 was 0.04 higher than that of ANFPSO4, and the mean MAE of LSSVR4 was 0.19 mm d^−1^ lower than that of ANFPSO4 (Fig. 4b). Models in the combination-based method had a mean NSE of LSSVR4 that was 0.07 higher than that of ANFPSO4 (Fig. 5). The results also show there was no significant difference in the RMSE between the LSSVR4 and ANFPSO4 models, but that the LSSVR4 model outperformed the ANFPSO4 one. These results confirm that combination-based LSSVR4 and ANFPSO4 were more accurate when calculating ET_ref_ than the other methods (Table 3).

The article "Comparison of predictions of daily evapotranspiration based on climate variables using different data mining and empirical methods in various climates of Iran" was retracted in 2026. Reasons: unreliable results or conclusions; concerns about the citations.

The mean NSE coefficients for the ML combination-based models in hyper-arid, arid, semi-arid and humid climates are 0.68, 0.74, 0.83 and 0.63, respectively. This indicates lower accuracy of the combination-based models for humid climates compared to arid and semi-arid ones (Fig. 5).

The estimated residual error range for daily ET_ref_ for all radiation-based models computed over a cumulative 12,053 days in hyper-arid, arid, semi-arid and humid climates were −4.8 to 11.4, −2.5 to 5.0, −1.1 to 2.6 and −1.1 to 1.3 mm d^−1^ in this order. The mean SI values for the mentioned climates were 0.18, 0.14, 0.12 and 0.15, respectively. Thus, it can be concluded that the lowest and highest accuracy of the combination-based models were linked to hyper-arid and semi-arid climates, respectively. In applied combination-based ML models, the LSSVR4 model had the highest R^2^ and the lowest RMSE. These results were predictable due to its reasonable inner model structure. The LSSVR4 is better in defining non-linear relationships between weather and ET_ref_ compared to other models, indicating a high performance as shown in Fig. 6.

The accuracy of the ET_ref_ estimation is based the SI. The best results among the 11 models were linked to the LSSVR4 model (Fig. 7) with the exception of Siri and Kish stations, where the SI value was more than 0.20. In other words, for 98% of the stations, the LSSVR4 model had estimated ET_ref_ values with good and excellent SI classifications (SI < 0.20). After the LSSVR4 model, the LSSVR3 and ANFPSO3 models had the highest accuracy by estimating the daily ET_ref_ values with good and excellent classifications for 93% of stations. The highest error among the studied models was related to the JEHA and PENM equations. About 90% and 76% of stations with poor classifications (SI > 0.30) were associated with the JEHA and PENM equations, respectively.

Among the empirical mathematical relationships, the BARO equation is most accurate with 79% of good and excellent classifications in estimating daily ET_ref_. The mean SI values for temperature-based, radiation-based, mass transfer-based and combination-based models for all studied stations are 0.17, 0.18, 0.14 and 0.13, respectively.

The mean SI was calculated as 0.35, 0.21, 0.19 and 0.23 for all studied models in the stations of hyper-arid, arid, semi-arid and humid climates, correspondingly. This indicates that most models err in estimating daily ET_ref_ in hyper-arid and humid climates and have their highest accuracy for semi-arid climates. Daily ET_ref_ estimations for stations located on the Persian Gulf (especially stations on the islands such as Siri, Kish and Abumusa) always had the highest errors. For example, the accuracies of estimating daily ET_ref_ on Siri Island by using all 11 SI models were always associated with the poor class (SI > 0.30). Most of the errors of the models at these stations depend on the greater complexity of the evapotranspiration process in arid and humid climates (Fig. 7).

The article "Comparison of predictions of daily evapotranspiration based on climate variables using different data mining and empirical methods in various climates of Iran" was retracted in 2026. Reasons: unreliable results or conclusions; concerns about the citations.

## 4 Conclusions and recommendations

According to the results, the behavior of the BARO equation was very good compared with complex models such as JEHA and PENM for different climates of Iran. However, it can be noted that empirical models are specific for the climatic conditions. Therefore, the BARO equation has an important role for stations without complete datasets and where it is not possible to utilize the PM-FAO_56_ equation or to develop ML models.

Temperature-based BARO and LSSVR1 significantly increased the accuracy of models used for predicting ET_ref_. Radiation-based LSSVR2 and ANFPSO2 models had higher precisions in predicting ET_ref_ than radiation-based JEHA equations. Mass transfer-based LSSVR3 and ANFPSO3 models performed significantly better than the radiation-based PENM equation. The performance and behavior of the combination-based LSSVR4 and ANFPSO4 models were similar to that of the combination-based empirical PM-FAO_56_ equation.

When combination-based models were available, all recommended ML models could assess ET_ref_ with a higher accuracy than empirical equations. The application of RH generally improved the performance for all climates, especially for the ML models. Although the role of RH can be more important for arid and semi-arid climates, this variable also provided performance gains for humid climates of Iran. Therefore, it can be recommended for future studies that the RH variable should be applied as a crucial parameter to predict ET_ref_ in humid climates. It is also recommended to analyze relationships between other meteorological variables and ET_ref_ and to apply other machine learning models including deep learning methods.

## Author contribution statement

Saeed Sharafi; Mehdi Ghaleni: Conceived and designed the experiments; Performed the experiments; Analyzed and interpreted the data; Contributed reagents, materials, analysis tools or data; Wrote the paper.

Miklas scholz: Conceived and designed the experiments; Analyzed and interpreted the data; Wrote the paper.

## Funding statement

This research did not receive any specific grant from funding agencies in the public, commercial, or not-for-profit sectors.

## Data availability statement

Data will be made available on request.

The article "Comparison of predictions of daily evapotranspiration based on climate variables using different data mining and empirical methods in various climates of Iran" was retracted in 2026. Reasons: unreliable results or conclusions; concerns about the citations.

## Declaration of interest's statement

.
